RETRACTED

# Optimization of Online Education and Teaching Evaluation System Based on GA-BP Neural Network

**DOI:** 10.1155/2021/8785127

**Published:** 2021-08-12

**Authors:** Xin Xu, Fenghu Liu

**Affiliations:** ^1^Undergraduate Academic Affairs Office, Shandong University of Arts, Jinan, Shandong 250000, China; ^2^Cavite State University, Don Severino de Las Alas Campus, Indang, Cavite 4100, Philippines; ^3^Wushu College, Shandong Sport University, Rizhao City, Shandong Province 276826, China

## Abstract

With the popularization and application of online education in the world, how to evaluate and analyze the classroom teaching effect through scientific methods has become one of the important teaching tasks in colleges. Based on this, this paper studies the application of the GA-BP neural network algorithm. Firstly, it gives a brief overview of the current situation of online education and GA-BP neural network algorithm. Secondly, through the investigation of the online education system in many aspects, it evaluates students' online education classroom teaching quality from five aspects, and this paper proposes a more scientific online education classroom teaching quality evaluation optimization model and finally verifies the reliability of the online education teaching evaluation model through the practice in a university. The results show that the GA-BP neural network-based evaluation optimization model can effectively evaluate the online education in the process of analyzing the quality of online education classroom teaching of most professional students.

## 1. Introduction

The current online education in colleges is mainly based on the traditional collective and group teaching, supplemented by the separate teaching of hierarchical teaching [1]. And, intelligence has become an important feature of the current online education classroom teaching system [2]. At present, the existing online education classroom teaching system provides a variety of methods, but it is difficult for students according to their own online education knowledge system architecture and examination knowledge focus [3]. The evaluation of classroom teaching quality in colleges and universities is relatively backward, and the research on it in some countries is relatively advanced [4]. Hu and Qin found that most of the online education still follow the traditional teaching ideas, ignoring the characteristics and differences of different students' online education ability, so the online education classroom teaching effect in colleges and universities cannot reach the optimal state [5]. Arciszewskl and Ziarko put forward an adaptive classroom teaching model of online education in colleges and universities based on multistrategy technology. Through the analysis of students' personality and online education advantages, different levels of classroom teaching can be carried out for different students, and hierarchical teaching can be realized in the teaching process [6]. Through experiments, Daniel et al. have proved that teaching methods can play a good role, effectively improve the effectiveness of online education classroom teaching, and use a number of indicators to evaluate students' online education ability [7]. Based on the traditional model theory and practical experience of online education, Ma et al. found that there is a problem of poor oral English in the current online education classroom teaching, so they proposed an adaptive teaching method based on the machine vision algorithm [8]. Through listening analysis of different online education dialogues, Gao et al. made students reach a state of deep thinking in the process of learning [9]. Chergui et al. proposed a new online education teaching method, analyzed the relationship degree of different modules in traditional online education classroom teaching, and established a multifactor coupling analysis model [10]. Smys et al. conducted a comprehensive evaluation on the selection of teaching forms, the classification of teaching contents, students' learning ability, etc., and adopted different students for experimental teaching [11]. The research results of Bibault et al. show that the online education teaching is better than the classical online education teaching method in obtaining heterogeneous information [12]. Curtu et al. put forward a hierarchical teaching method based on online pedagogy theory through different students [13]. Lucas et al. have verified it through teaching practice. The final results show that it is suitable for the teaching planning of online education and for finding the optimal teaching scheme [14]. Alarifi et al. proposed a new group online education and teaching method based on hyperchaotic mapping, which used the transformed chaotic sequence to scramble the position of the original online method, and realized the optimal determination of various teaching methods in the process of online education classroom teaching in colleges and universities [15]. The results of Constantin et al. show that the teaching scheme of group online education in colleges and universities has good teaching effect, which is suitable for the online education of junior and senior students [16]. To sum up, it can be seen that most of the current online education classroom teaching modes in colleges and universities do not involve the intelligent algorithm based on the difference of the characteristics of the student group [17]. There are relatively few research results on specific quantitative dynamic evaluation system and quality evaluation of online education classroom teaching [18]. And, there is no research on the objectivity of online education in colleges and universities and the construction of relevant models [19, 20].

RETRACTED

In this context, this paper proposes a GA-BP neural network algorithm-based online education classroom teaching quality evaluation optimization model. The local clustering algorithm based on high degree of relationship and double correlation factors is selected, and three characteristic parameters related to the online education classroom teaching mode and teaching effect influence index are adopted. An online education classroom teaching evaluation system based on the local clustering algorithm is proposed. Through the research of the online teaching process, the hierarchical framework and index relationship of the whole online education classroom teaching system are clearly defined. This paper evaluates the system from multiple perspectives and provides a comprehensive index for the quality evaluation of the online education classroom teaching system. Then, it uses the GA-BP neural network algorithm to analyze the characteristics of the online education classroom teaching effect. This study is divided into three parts. The first part introduces the research status of influencing factors of online education classroom teaching effect. The second part constructs the online education classroom teaching evaluation model based on GA-BP and constructs the online education classroom teaching quality evaluation index system by using the Laplace factor method. The third part verifies the relevant indicators of the online education classroom teaching evaluation model and draws a conclusion.

## 2. GA-BP Neural Network Algorithm and Basic Idea in Online Teaching Quality Evaluation Model

GA-BP neural network algorithm is a common algorithm for effectively extracting and discovering the correlation degree between different data. On the contrary, the GA-BP neural network algorithm has become a hot research topic in many fields such as information mining and target content retrieval. It is to solve the problem of “divide the target dataset into multiple groups according to certain rules.” Generally speaking, it is the process of classifying the highly correlated group into one group and the less correlated group. The GA-BP neural network algorithm is also a basic method of self mining [21]. The GA-BP neural network algorithm is used to cluster the target. Its more application fields are to detect the information association and match of the target object or to search and screen unknown targets in the fuzzy way. In order to realize the data mining under this algorithm, the target data information should be translated into the language information recognized by the computer through certain patterns [22–24]. In general, relevant technicians will use the vector space model to process the feature data of the target object in an information-based way. The GA-BP neural network algorithm is a common data mining and information training algorithm [25].

RETRACTED

This study applies the GA-BP neural network algorithm to the evaluation of online education teaching quality. On this basis, the study can make full use of the learning data and test results of each student in online education class and realize the overall approach by tracking dynamically in real time. The similarity degree and the preperiod index of each comparison column and reference column can be quantitatively described by local correlation factors. The quantitative index is used to sort the influence degree of the online education classroom teaching index, which can effectively analyze the factors affecting the quality of online education classroom teaching.

### 2.1. Optimization Model of Online Education Classroom Teaching Quality Evaluation Based on GA-BP Neural Network Algorithm

#### 2.1.1. The Construction Process of Classroom Teaching Quality Evaluation Model of Online Education in Colleges and Universities

In order to realize the scientific analysis of the teaching quality of online education, this paper takes the students of most majors in colleges and universities as the basic research objects, investigates the different aspects of the students of most majors in colleges and universities, then analyzes these data, and finally evaluates the online education ability of the research objects. This is also the basic realization process of the investigation and research on the online education ability of most college students. The content types of the research are shown in Table 1.

The specific model construction process is as follows.

First of all, the online education level of most professional students in the target university is the first survey data (mainly the score records of online education courses), and the relevant system will extract the characteristic information of the data and then carry out computer language processing to convert it into binary number so that the computer can store and compare with the existing database information. The data acquisition and training process are shown in Figure 1.

Secondly, we issue some research questions to the investigated subjects, summarize the options of different research objectives through different options (A/B/C/D), so as to form the second research data, and then input the options into the computer system, The computer's database information and preset automatic judgment program (mainly based on the psychological analysis behind different options) can restore some data information, so as to realize the reprocessing and reciprocating cycle of the first data and the second data information. The data analysis process is shown in Figure 2.

RETRACTED

Finally, it is targeted to delete or remove some irrelevant or meaningless data information and record by vector to form a special data information record, which realizes the transformation of data information into vector information, and in and out of storage. For the calculation and recognition of similarity, the computer calculates the distance and angle between different vectors. The closer the distance or the smaller the angle, the higher the similarity of the data information contained in the two vectors and the higher the positive relationship between the theoretical knowledge of online education and the actual level of online education of most college students. The judgment and classification process is shown in Figure 3.

Let *x*_*i*_=(*x*_*i*1_, *x*_*i*2_,…, *x*_*ip*_) and *x*_*j*_=(*x*_*j*1_, *x*_*j*2_,…, *x*_*jp*_) be the observed values of *i* and *j* targets; then, the similarity measure *δ*_*ij*_ between them is

(1) $$\begin{array}{c} \delta_{ij}=\frac{\sum_{k=1}^{p}\left(x_{ik}-{\bar{x}}_{i}\right)\left(x_{jk}-{\bar{x}}_{j}\right)}{i+j}. \end{array}$$

The corresponding coupling degree judgment formula *c*_*ij*_ is as follows:

(2) $$\begin{array}{c} c_{ij}=\underset{n⟶\infty }{\lim}\frac{\sum_{k=1}^{n}x_{ki}x_{kj}}{\sqrt{\sum_{k=1}^{n}x_{ki}^{2}\sum_{k=1}^{n}x_{kj}^{2}}}. \end{array}$$

The correction coefficient *Q*_*ij*_ is

(3) $$\begin{array}{c} Q_{ij}=\sqrt{1-c_{ij}^{2}}. \end{array}$$

The sum of squares coefficient *s*_1_^2^ is

(4) $$\begin{array}{c} s_{1}^{2}=\underset{n⟶\infty }{\lim}\frac{1}{n}{\sum_{k=1}^{n}\left[x^{\left(0\right)}k-{\bar{x}}^{\left(0\right)}\left(k\right)\right]}^{2}. \end{array}$$

The average coefficient ${\bar{x}}^{\left(n\right)}\left(k\right)$ under the reciprocal of order *k* and the operation value $\bar{e}\left(k\right)$ between different clusters are as follows:

(5) $$\begin{array}{c} {\bar{x}}^{\left(n\right)}\left(k\right)=\underset{n⟶\infty }{\lim}\frac{1}{n}\sum_{k=1}^{n}x^{\left(n\right)}\left(k\right), \end{array}$$

(6) $$\begin{array}{c} \bar{e}\left(k\right)=\underset{n⟶\infty }{\lim}\frac{1}{n}\sum_{k=1}^{n}e\left(k\right), \end{array}$$

where *s*_1_^2^ is the weighted sum of square differences, *x*^(0)^*k* is the vector to be detected within the cluster, ${\bar{x}}^{\left(0\right)}\left(k\right)$ is the standard reference vector within the cluster, ${\bar{x}}^{\left(n\right)}\left(k\right)$ is the average value processed between different clusters, *x*^(*n*)^*k* is the vector processing value between different clusters, $\bar{e}\left(k\right)$ is the operation value between different clusters, and *e*(*k*) is the processing value within each cluster.

RETRACTED

#### 2.1.2. Application of BP Neural Network Algorithm in Online Education Teaching Evaluation Model of Colleges and Universities

The BP neural network algorithm used in this evaluation model has many advantages. For example, in the process of analyzing and investigating the current situation of online education ability of college students, through the comparative analysis of the results of online education theory courses and questionnaire data of most college students, and then after processing these two kinds of big datasets, the algorithm can be scalable and efficient, and the algorithm will end with local optimization. The BP neural network algorithm also has some shortcomings in the process of dealing with the online education quality evaluation of college students of different majors. The degree of data processing in different questionnaires is not uniform. On the contrary, the BP neural network algorithm requires users to give the number of clusters to be generated in advance during the data analysis of the questionnaire. The training process from initial to multiple adaptive coupling is shown in Figure 4.

Finally, because the BP neural network algorithm is sensitive to the initial value of the dataset, for different initial values of the questionnaire (that is, the data options in the first question of the questionnaire will affect the evaluation effect of the follow-up questionnaire), this may lead to different data analysis results.

#### 2.1.3. Improvement Strategy of GA-BP Neural Network Algorithm

In view of the problems of the BP neural network algorithm, we make some improvements to the intelligent data mining algorithm (GA-BP neural network algorithm).

In the first step, in the questionnaire survey data of *n* targets, multiple target data are determined irregularly as the center of the initial clustering data set and compared with the second target vector which needs to be detected. The calculation formula of disturbance adaptive degree *D*_*tr*_^2^ is as follows:

(7) $$\begin{array}{c} D_{tr}^{2}=\frac{n_{l}}{n_{r}}{\bar{x}}^{2}\left(k\right), \end{array}$$

where *n*_*l*_ and *n*_*r*_ are fitness index values and satisfy the following relationship:

(8) $$\begin{array}{c} n_{l}+n_{r}=n_{m}, \end{array}$$

where *n*_*m*_ is the index value of the target vector.

RETRACTED

The second step is to put the questionnaire survey data and online education theory knowledge data of other target students into the set closest to the initial data according to the setting and comparison of multiple parameter values in a random way or sorting order to form the first cluster and calculate and transform the distance between the vectors of different clusters to realize the average connection between groups and the average connection within groups. The discriminating function *w*(*x*) is

(9) $$\begin{array}{c} w\left(x\right)=\frac{x_{1}+\cdots +x_{n}}{n^{2}}, \end{array}$$

where *x*_1_+⋯+*x*_*n*_ is the sum of all samples and *n* is the total number of samples.

The third step is to redetermine the sample center of each neural network training link and determine the spatial vector of the initial cluster students' online education theory course data. Then, according to the shortest distance comparison of different categories, determine the similarity arrangement between different clusters, and form a cluster group with the logical structure. The cluster group correction function *H*(*x*) is

(10) $$\begin{array}{c} H\left(x\right)=w^{2}\left(x\right)\underset{n⟶\infty }{\lim}\frac{\sum_{i=1}^{\infty }x_{i}^{2}}{n+1}. \end{array}$$

In the fourth step, after repeating the second and third steps, when the last group of online education classroom teaching quality evaluation questionnaire data and students' online education performance data are input, the processing and classification of this group of data information are realized, and the next group of data information is judged again. Then, the feature items of different clusters are weighted, and the square difference is calculated. The similarity of data information between clusters is based on the average value and compared with the preset standard value to achieve secondary verification so as to distinguish the best and find out the best comprehensive solution. The simulation training results are shown in Figure 5. As can be seen from Figure 5, the GA-BP neural network algorithm has a higher degree of agreement than the BP neural network algorithm and conventional neural network algorithm, and the lowest degree of agreement can also reach 0.969, so its optimization effect is more obvious.

## 3. Result Analysis and Discussion

### 3.1. Practice Test Process of Classroom Teaching Innovation Model of College Online Education Based on GA-BP Neural Network Algorithm

In order to find the relevance between the online education level and the online education classroom teaching quality of different students in colleges and universities as well as the relevance between the academic performance of most professional students and the online education classroom teaching, the practical test is carried out based on the online education examination data of the actual students in a university. This time, the improved GA-BP neural network algorithm is adopted. According to different parameter settings, it will divide the target students' academic performance information and online education classroom teaching data into multiple training centers. Through the comparative analysis of different parameters and the comparative analysis of the distance and angle between the relevant data and information converted into the space vector, ensure that each cluster has a high degree of similarity and data information matching rate. The objective evaluation criteria of the online education teaching evaluation system during the experiment are shown in Table 2.

RETRACTED

The error analysis of experimental results obtained by GA-BP, BP, and traditional neural network algorithm (TNN) is shown in Figure 6.

It can be seen from Table 2 and Figure 6 that, in the online education teaching evaluation system, with the increase of training times, the error is smaller and smaller because the GA-BP neural network algorithm can use multiple target data as the initial clustering dataset center point and compare with the second target vector to be detected by comparing the distance between them. Then, by calculating the angle and distance between different vectors and comparing with the set value, we can know the similarity between the data information represented by the target vector and the reference data, so as to realize the judgment of the similarity. Then, according to the shortest distance comparison of different clusters, the similarity arrangement between different clusters is determined to form a cluster group with the logical structure. Finally, due to the actual questionnaire data, the number of outliers of different questions is often unpredictable. For example, in this research, in the questionnaire data of online education classroom teaching quality of most college students, the learning objectives of the same question with the same options are summarized, and then, the college student groups are analyzed after the summary and classification. In this way, the influence of sample input order on the selection of initial clustering center is reduced, so as to improve the efficiency of the whole data mining algorithm for data analysis.

### 3.2. Experimental Results and Analysis of Online Teaching Evaluation System

The experimental comparison method (experimental group and control group) have been carried out in the following ways: one-to-one offline survey, random paper survey, and online evaluation system survey. The subjects of the survey are college students of most majors in a university. For different genders of college students, we use different ways of questionnaire survey content. The questionnaire includes the following aspects: online education oral ability, online education writing ability, online education reading ability, classroom student participation, homework completion, class average score, etc. In the process of this survey, we systematically distributed 400 questionnaires to the students of most majors in our university through the support of a university and effectively recovered 399 questionnaires, including 197 for boys and 202 for girls. The proportion of male and female participants in the experiment is shown in Table 3.

RETRACTED

The specific experimental data of online education classroom teaching quality evaluation are shown in Table 4.

The satisfaction results of different numbers of students (50, 100, 200, 300, and 400) to the online education teaching evaluation system are shown in Figure 7.

It can be seen from Tables 3 and 4 and Figure 7 that, through this experiment and research, in the online education classroom teaching process of most majors in colleges and universities, the overall teaching quality is relatively good. Among the overall respondents, 91.3% of the students are satisfied with online education classroom teaching, among which 32.2% are female students and 59.1% are male students. In these online education examinations, 89.3% of the people had obvious effect improvement, among which 61% were girls and 39% were boys. When it comes to specific online education module knowledge, such as writing, reading, and online teaching interaction, 86.1% of the people clearly improve this aspect. When it comes to online classroom participation, such as students actively answering teachers' questions, 48.8% of the students actively participate in this link, that is, almost half of the students rarely participate in classroom *Q* and *A*. When asked whether the online education teaching method is effective, 86.0% of the college students surveyed agree with the teacher's teaching method. Although the dataset used in the training model in this experiment is randomly processed during the acquisition process, it still has a certain degree of impact on the reliability of the experimental results, so this research is in the above experimental process carried out no less than 30 repetitive experiments and took the average value, so it has strong universality and authenticity in the reliability of the experimental results.

RETRACTED

## 4. Conclusion

The traditional classroom online education in colleges cannot meet the current objective requirements. Based on this, this paper studies the classroom teaching quality evaluation model of online education in colleges based on the GA-BP neural network algorithm. Firstly, the research status of online teaching quality evaluation of college students and GA-BP neural network algorithm are briefly summarized. Then, according to the five factors that affect the evaluation of online education, a new evaluation method is proposed, and a more scientific online education teaching quality evaluation model is constructed. Finally, through the practice in a university, the reliability of the online education classroom teaching quality evaluation model is verified. The research results show that, in the process of analyzing the teaching effect of online education for most college students, the method based on the GA-BP neural network algorithm cannot only effectively evaluate the teaching effect but also can be used to analyze and evaluate the current situation of college students' online education ability. However, this paper only focuses on the construction of online education teaching evaluation model and data clustering and does not consider how to strengthen the local focus of the evaluation system. Therefore, before the implementation of online education in colleges, we can make in-depth research from the local factors' variable weight of the system.

## Figures and Tables

**Figure 1:** Data acquisition and training process of online teaching.

**Figure 2:** Data analysis process of online teaching.

**Figure 3:** Data relevance judgment classification process.

**Figure 4:** Adaptive training process of the BP neural network model.

**Figure 5:** Simulation training results under different neural network methods.

**Figure 6:** Error analysis of the improved experimental results.

**Figure 7:** Different numbers of students' satisfaction with online education and teaching.

**Table 1:** Survey content of the online education ability status.

Investigate subject	Number of people participating in the survey
Self-study ability	400
Communication skills	396
Interactive ability	400
Teamwork ability	398
Application innovation ability	392
Language skills	395

**Table 2:** Objective evaluation standards for online education and teaching systems.

Objective evaluation criteria	Evaluation level
Topic relevance	A/B/C/D/E
Explain logic	0–10
Teacher-student interaction	A/B/C/D/E
Online *Q* and *A* effect	A/B/C/D/E
Online classroom task completion	0–10

**Table 3:** Ratio of men and women participating in the experiment.

The total number of questionnaires	400
The total number of boys in the survey	197
The total number of girls in the survey	202

RETRACTED

**Table 4:** Experimental data of online education classroom teaching quality evaluation.

Experimental evaluation data	Percentage (%)
Student satisfaction with online teaching	91.3
People who have noticeably improved the test process	89.3
People with significant improvement in writing and other processes	86.1
Number of active participants	48.8
People who recognize teaching methods	86.0
Compared with the current mainstream intelligent online education classroom (NN model), the teaching quality has improved	29.3

## Data Availability

The data used to support the findings of this study are available from the corresponding author upon request.
